# Study on the Killing Effect of *γδ*T Cells Activated by Rukangyin on Breast Cancer MDA-MB-231 Cells

This article has been retracted.

**DOI:** 10.1155/2021/5838582

**Published:** 2021-10-15

**Authors:** Zaiwang Chen, Yujuan Zhao, Xiangqi Li, Keqiang Wang

**Affiliations:** ^1^Department of Laboratory Medicine, Second Affiliated Hospital of Shandong First Medical University, Tai'an, Shandong Province, China 271000; ^2^Department of Laboratory Medicine, Shan County Central Hospital, Shan County, Shandong Province, China 274300; ^3^Department of Emergency Medicine, Yingsheng District, Tai'an Central Hospital, Tai'an City, Shandong Province, China 271000; ^4^Breast Surgery, Second Affiliated Hospital of Shandong First Medical University, Tai'an, Shandong Province, China 271000

## Abstract

**Objective:**

To investigate the killing effect of rukangyin (RKY) activated *γδ*T cells on breast cancer cells MDA-MB-231 and to provide a basis for Chinese medicine combined with immunotherapy for breast cancer.

**Methods:**

Thus, study isolates peripheral blood mononuclear cells (PBMC) and uses CCK8 to select the optimal concentration of Rukang drink, ZOL (zoledronic acid), and PHA (phytoagglutinin) to activate *γδ*T cells. There are 8 groups including the ① PBMC control group, ② RKY group, ③ ZOL group, ④ PHA group, ⑤RKY+ZOL group, ⑥RKY+PHA group, ⑦ZOL+PHA group, and ⑧ RKY+ZOL+PHA group. At 0 and 14 days of culture, cell viability and *γδ*T cell expansion were detected by flow cytometry. The 8 groups of amplified *γδ*T were cocultured with breast cancer MDA-MB-231 cells labeled with fluorescent dye CFSE at a ratio of 10 : 1 to determine the lethality of *γδ*T cells on breast cancer MDA-MB-231 cells.

**Results:**

The optimal concentrations of RKY, ZOL, and PHA to activate *γδ*T cell proliferation were 4.5 mg/l, 3 *μ*M, and 60 *μ*g/ml, respectively. On day 0 of culture, the values ($\bar{x}\pm s$, %) of *γδ*T cells in groups ① to ⑧ were 3.50 ± 0.72, 3.97 ± 0.45, 3.99 ± 0.15, 4.37 ± 0.24, 4.47 ± 0.97, 4.59 ± 1.35, 3.45 ± 0.40, and 3.89 ± 0.48, while when a comparison between groups was made, *F* = 1.093 and *p* = 0.412; there is no significant difference between groups. Besides, when being cultured for 14 days, the values ($\bar{x}\pm s$, %) of *γδ*T cells in groups ① to ⑧ were 4.77 ± 0.78, 23.22 ± 2.73, 26.4 ± 0.92, 28.66 ± 1.43, 27.99 ± 1.10, 30.21 ± 1.91, 32.51 ± 0.74, and 33.21 ± 0.42. Then, based on the comparison between groups, *F* = 119.917 and *p* < 0.001, there are obvious statistical differences between groups. Furthermore, the expansion values of *γδ*T cells were compared before and after culture for 0 and 14 days. The *t* values of group ① to group ⑧ were 2.072, 12.051, 41.641, 29.015, 27.777, 18.972, 59.836, and 79.622. Except for the PBMC control group (*p* = 0.107), there are significant statistical differences (*p* < 0.001). The number of *γδ*T cell expansion at 14 days was the RKY+ZOL+PHA group>ZOL+PHA group>RKY+PHA group>PHA group>RKY+ZOL group>ZOL group>RKY group>PBMC control group. From group ① to group ⑧, the *γδ*T cell expansion multiples were 1.14 ± 0.44, 5.25 ± 0.77, 5.70 ± 0.89, 6.05 ± 1.03, 6.21 ± 0.09, 6.76 ± 1.46, 7.52 ± 1.05, and 7.97 ± 1.55, respectively, while the comparison between groups was *F* = 17.772 and *p* < 0.001. As for the amplification factor, there was RKY+ZOL+PHA group>ZOL+PHA group>RKY+PHA group>RKY+ZOL group>PHA group>ZOL group>RKY group>PBMC control group. In the killing experiment, the killing rate ($\bar{x}\pm s$, %) of group ① to group ⑧ was 1.08 ± 0.03, 1.89 ± 0.14, 1.22 ± 0.11, 1.31 ± 0.09, 1.48 ± 0.10, 2.02 ± 0.21, 2.18 ± 0.27, and 2.37 ± 0.35, whereas the comparison between groups was *F* = 20.498 and *p* < 0.001. In terms of killing rate, there was RKY+ZOL+PHA group>ZOL+PHA group>RKY+PHA group>RKY group>RKY+ZOL group>PHA group>ZOL group>PBMC control group.

**Conclusion:**

Rukangyin can increase the lethality of *γδ*T cells against MDA-MB-231 cells by activating the proliferation of *γδ*T cells, which provides a basis for Chinese medicine combined with immunotherapy for breast cancer.

## 1. Introduction

Breast cancer, as the most common malignant tumor, seriously threatens women's health and even lives. The incidence of triple-negative breast cancer (TNBC, ER, PR, and HER-2 are all negative) accounts for approximately 15%-20% of breast cancer. Breast cancer has the highest mortality and the worst prognosis. Traditional treatment methods mainly include surgery, radiotherapy and chemotherapy, endocrine therapy, and targeted therapy. However, a large number of patients still have metastasis or recurrence, which may be associated with the immune system such as tumor resistance, oncogene activation, and cellular pathway activation. Our previous studies have shown that Rukang decoction (the main active ingredients are saikosaponin A (C_42_H_68_O_13_), curcumol (C_15_H_24_O_2_), pachymic acid (C_33_H_52_O_5_), astragaloside-II (C_43_H_70_O_15_), hesperidin (C_28_H_34_O_15_), coixenolide (C_38_H_70_O_4_)) can inhibit the proliferation and induce apoptosis of triple-negative breast cancer cells MDA-MB-231, verifying that the compound Chinese medicine has the therapeutic effect of soothing the liver and spleen on the treatment of breast cancer [1–4]. T cells are divided into *αβ*T cells and *γδ*T cells in accordance with different TCR types. *γδ*T cells account for only 0.5 to 5% of adult peripheral blood [5, 6], which are mainly distributed in mucosa and subcutaneous tissues and dominate an important role in antimicrobial, parasite, and tumor immunity [7–13]. In this study, rukangyin (RKY), zoledronic acid (ZOL), and phytohemagglutinin (PHA) of appropriate concentrations were used as stimulants to act on PBMC. In addition, the induced and proliferated *γδ*T cells were collected as effector cells. Human breast cancer cell line MDA-MB-231 was used as the target cell to observe the killing effect of proliferated *γδ*T cells on breast cancer cell line MDA-MB-231, aiming to explore the use of rukangyin to induce and activate *γδ*T cells in breast cancer immunotherapy applications.

## 2. Materials and Methods

### 2.1. Materials and Methods

#### 2.1.1. Experimental Materials and Equipment

MDA-MB-231 cells (Sai Baikang, article number: Icell-h133), Rukang drink (homemade), ZOL (MCE, article number: HY-13777A), PHA (MCE, article number: HY-N7038), human peripheral blood lymphocyte separation solution (Solarbio, article number: P8610), CFSE (MCE, article number: HY-D0938), TCR *γ*/*δ* PE (Biolegend, article number: 331209), CD3 PerCP (Biolegend, article number: 300325), CCK8 detection kit (KEYGEN, article number: KGA317), R1640 complete medium (ScilenCell, article number: 1001), D trypsin-ETA digestion solution (Solarbio, article number: T1300), PBS (BI, article number: 02-024-1ACS), green chain mycin mixture (100x) (Solarbio, article number: P1400), FBS (BBI Life Sciences, article number: E600001-0500), DMEM complete medium (KGM, article number: KGM12800S-500) were used. NovoCyte™ flow cytometer (Aisen Biotech (Hangzhou) Co., Ltd., model: NovoCyte 2060R) and CO_2_ incubator (Shanghai Yiheng Scientific Instrument Co., Ltd., model: BPN-80CW) were used.

#### 2.1.2. Preparation of Main Reagents

(1) For Rukang Yin, we add 100 ml of distilled water for boiling 9 g of each medicine package, fully dissolve and filter; pour 100 ml of sterilized distilled water to dilute and filter for preparing a solution with a concentration of 45 mg/ml; and then dilute according to the needs of the experiment. (2) For ZOL, we accurately weigh 3.5 mg, add 3.5 ml of PBS for dissolving it, prepare a solution with a concentration of 3.45 mM, and dilute it according to experimental needs. (3) For PHA, 5 mg is precisely added to 1 ml of PBS to dissolve it. Then, it will be prepared into a solution with a concentration of 5 mg/ml and diluted according to the needs of the experiment. (4) For CFSE, 10 mg is precisely added to 1 ml of DMSO solution to prepare a solution with a concentration of 17.9385 mM and diluted according to actual needs

### 2.2. Method

#### 2.2.1. Separation of PBMC

The current study was performed according to the Declaration of Helsinki and was approved by the ethics committee of the Second Affiliated Hospital of Shandong First Medical University. In the morning, fresh peripheral blood was drawn from healthy volunteers on an empty stomach and diluted 1 : 1 with phosphate-buffered saline (PBS). Moreover, PBMCs were separated in line with Ficoll density gradient centrifugation for use.

#### 2.2.2. CCK8 Detects Cell Proliferation and Screens Drug Concentration

(1) The digested cells were resuspended and counted. Different concentrations of drugs were grouped and plated, and the cell density was 1 × 10^4^/well. (2) After 24 hours of cell growth, we replace the 96-well plate cells to be tested with the same medium, with 100 *μ*l per well, add 10 *μ*l CCK8 reagents to each well, and incubate in an incubator for 2 hours. (3) The microplate reader detects the absorbance of each well at 450 nm wavelength. According to cell proliferation, the optimal concentration of rukangyin, ZOL, and PHA to activate *γδ*T cells was screened out. There are 8 groups including the ① PBMC control group, ② RKY group, ③ ZOL group, ④ PHA group, ⑤ RKY+ZOL group, ⑥ RKY+PHA group, ⑦ ZOL+PHA group, and ⑧ RKY+ZOL+PHA group, which were tested after 14 days of culture

#### 2.2.3. Test Cell Viability with Trypan Blue

According to the principle that the trypan blue dye cannot enter cells with intact cell membranes, it can only accumulate in cells with damaged or dead cell membranes and present blue under the microscope for cell viability statistics. The steps are listed as follows: (1) collect the cell liquid, centrifuge, discard the supernatant, add thefresh medium for resuspending, count, and prepare a single-cell suspension and (2) mix the cell suspension with 0.4% trypan blue solution at a ratio of 9 : 1. Within three minutes, we count live and dead cells under a microscope. After that, dead cells can be stained blue, while live cells are not. Statistics of cell viability can be calculated as follows: living cell rate (%) = total number of live cells/(total number of live cells + total number of dead cells).

#### 2.2.4. Flow Cytometric Detection of *γδ*T Cell Expansion Times

(1) We collected 1 × 10^6^-3 × 10^6^ cells, centrifuge to remove the supernatant, add 1 ml PBS for washing once at 1500 rpm and centrifuging for 5 min, and finally, discard the supernatant. (2) We add 50 *μ*l PBS for resuspending the cells and add 5 *μ*l antibody TCR *γ*/*δ* PE and CD3 PerCP, respectively. After lightly mixing, we incubate at room temperature for 20 minutes in the dark. (3) We add 1 ml PBS, centrifuge at 500 rpm for 5 min, and discard the supernatant; we add 500 *μ*l PBS for resuspending the cells, mix well, and check the amplification factor on the flow meter: Amplification factor = (total number of cells after amplification × *γδ*T cells after amplification Purity)/(Total cell number before expansion × *γδ*T cell purity before expansion).

#### 2.2.5. Recovery of Breast cancer MDA-MB-231 Cells

(1) We puted the prepared culture medium required for cell recovery in a dry constant temperature heater at the temperature of 39°C and preheat for half an hour. (2) We removed the cells to be recovered from liquid nitrogen and transfer them through a dry ice box. Then, the cells were put into the dry-type constant temperature heater and quickly placed into the ultraclean table after thawing. (3) The cells were transferred to the centrifuge tube, marked and centrifuged (1000 rpm, 3 min), and discarded the supernatant. (4) The fresh medium was added to the centrifuge tube to resuspend the cells, transferred to a cell culture flask, and placed in a 37°C, 5% CO_2_ incubator to continue culturing.

#### 2.2.6. Flow Cytometric Detection of *γδ*T Cell Killing Rate

The amplified PBMCs from group ① to group ⑧ were cocultured with breast cancer MDA-MB-231 cells labeled with fluorescent dye CFSE at a ratio of 10 : 1. After washing with PBS, the cells were resuspended and added 7-AAD for avoiding light. After 15 minutes of incubation, flow cytometry was used to determine the lethality of *γδ*T cells on breast cancer MDA-MB-231 cells: cell killing rate (%) = [experimental group (CFSE + 7 − AAD+/CFSE+) − control group (CFSE + 7 − AAD+/CFSE+)] × 100%.

#### 2.2.7. Statistical Analysis

All data were statistically analyzed by SPSS19.0. Significant differences were determined by SPSS one-way analysis of variance. In addition, *p* < 0.05 was regarded as the significant difference.

## 3. Result

### 3.1. Drug Concentration Screening

Under different drug concentrations, according to the proliferation of *γδ*T cells, the optimal rukangyin concentration is 4.5 mg/l, ZOL concentration is 3 *μ*M, and PHA concentration is 60 *μ*g/ml.

### 3.2. Trypan Blue to Detect Cell Viability

PBMCs in each group were counted by trypan blue staining on day 0 and day 14. The results are shown in Table 1 and Figures 1 and 2. Before PBMC was added to the drug culture, the cell viability was 100%, and the condition was good. After 14 days of adding the drug, the cell viability of each group was above 90% with good condition.

### 3.3. Flow Cytometric Detection of *γδ*T Cell Expansion Times

From group ① to group ⑧, the expansion results of *γδ* T cells on day 0 and day 14 of culture are shown in Table 2 and Figures 3–5. When cultured for 0 days, *γδ*T cell values were compared between groups (*F* = 1.093, *p* = 0.412), and there existed no significant difference between the groups. When cultured for 14 days, the *γδ*T cell values were compared between the groups (*F* = 119.917, *p* < 0.001). In addition, there were significant statistical differences between the groups. *γδ* T cell expansion value was RKY+ZOL+PHA group>ZOL+PHA group>RKY+PHA group>PHA group>RKY+ZOL group>ZOL group>RKY group>PBMC control group. The comparison of the *γδ*T cell expansion values before and after the growth of *γδ*T cells at day 0 and day 14 in each group showed significant statistical differences except for the PBMC control group. After 14 days of culture, the expansion multiples of *γδ*T cells in each group are shown in Table 3 and Figure 6. The ratio between each group was *F* = 17.772, *p* < 0.001, and there existed a significant difference. Compared with the control group, the amplification factor of each group increased and the amplification factor was RKY+ZOL+PHA group>ZOL+PHA group>RKY+PHA group>RKY+ZOL group>PHA group>ZOL group>RKY group>PBMC control group.

### 3.4. Flow Cytometric Detection of *γδ*T Cell Killing Rate

From group ① to group ⑧+MDA-MB-231 cells, the killing results are shown in Table 4 and Figures 7–9. Based on comparison between groups (*F* = 20.498, *p* < 0.001). Significant differences can be found. Killing rate was RKY+ZOL+PHA group>ZOL+PHA group>RKY+PHA group>RKY group>RKY+ZOL group>PHA group>ZOL group>PBMC control group.

## 4. Discussion

Breast cancer is regarded as the most common malignant tumor in women. TNBC is a pathological subtype of breast cancer. Due to the lack of appropriate endocrine and targeted therapy drugs, only surgery, radiotherapy, and chemotherapy are currently recommended as the main treatment methods [14]. Immunotherapy is an emerging tumor treatment model following surgery, radiotherapy, and chemotherapy. It stimulates or modulates the body's immune system to enhance the tumor microenvironment's antitumor immunity, thus controlling and killing tumor cells. Therefore, it is expected to become an innovation in the field of tumor therapy. The presence of tumor antigens is a prerequisite for antigen-specific T cell activation. The tumor mutation burden varies significantly among different subtypes of breast cancer, among which TNBC has the highest mutation burden [15]. *γδ*T cells are T cell antigen receptors (T cell receptor (TCR)). T cells composed of *γ* and *δ* chains. They are extensively distributed in peripheral blood and mucosal tissues of the body [16]. They are connected to natural immunity and adaptation in antitumor immunity. Activated *γδ*T cells can exert their cytotoxic effects on tumor cells through a variety of ways and have good antitumor effects both in vivo and in vitro [17]. *γδ*T cell immunotherapy technology, as a new tumor therapy, has good application prospect.

Activated *γδ*T cells have a direct killing effect on tumor cells. Their cytotoxicity is similar to CD8+ cytotoxic T cells and NK cells. They can secrete perforin and granzyme B to destroy cell membranes or express apoptosis-inducing factors, such as CD95 ligand and TNF-related apoptosis-inducing ligand (TRAIL) kill tumor cells [18]. In view of the multiple antitumor mechanisms of *γδ*T cells, people are adopting two strategies to use *γδ*T cells for tumor immunotherapy: isolation and in vitro expansion of V*γ*9V*δ*2 T cells, adoptively infused into patients and/or in vivo application of V*γ*9V*δ*2 such as the zoledronic acid T cell activator for enhancing the antitumor activity of *γδ*T cells. Besides, there are two methods for adoptive infusion of *γδ*T cells: one is to collect peripheral blood mononuclear cells (PBMC) from tumor patients, isolate *γδ*T cells, use NBPs and IL-2 to amplify and activate them, and then return them to the patient, or in other words, the antitumor activity of *γδ*T cells is used to treat tumors, while the second is to collect PBMC from tumor patients to isolate *αβ*T cells, transfer TCR*γδ* DNA into *αβ*T cells, and make *αβ*T cells express TCR*γδ*, thus being amplified in vitro and then infused back to the patient [19]. Our research group used Mycobacterium tuberculosis low-molecular-weight polypeptide antigen (Mtb-Ag) to amplify and activate *γδ*T cells and can quickly obtain sufficient *γδ*T cells [5].

Previously, RKY inhibited breast cancer lymphatic metastasis and played a certain role in breast cancer treatment by regulating PI3K/AKT and other signaling pathways, inhibiting breast cancer cell proliferation, and inducing apoptosis [1, 2]. According to the present study, RKY, PHA, and ZOL can stimulate the proliferation of *γδ*T cells at appropriate concentrations. CCK8 was employed to detect the proliferation of PBMC at different concentrations of RKY. It was screened out that when the RKY concentration was 4.5 mg/l, the proliferation of PBMC was the highest. PHA is a mixture of glycoprotein and protein extracted from plants. It can cause the agglutination of red blood cells and obtain its name. It can also stimulate the proliferation of PBMC [20]. In the present study, the PHA concentration was between 0 and 60 *μ*g/ml, and the proliferation of PBMC was the highest at 60 *μ*g/ml. With the increase of PHA concentration, the cell proliferation rate gradually increased, which is consistent with the report of Wang et al. [21]. ZOL is a third-generation bisphosphonate drug. It is a drugwhich can be used to treat osteoporosis and tumor bone metastasis. Its application in the proliferation of *γδ*T has been reported in numerous reports [22, 23]. In the current experiment, CCK8 was used to detect the proliferation of monocytes with different concentrations of ZOL. Moreover, it was screened out that the cell proliferation rate of ZOL reached the maximum at a concentration of 3 *μ*M. From 0 to 20 *μ*M, as the concentration of ZOL increases, the proliferation rate of monocytes increases first and decreases at high concentrations. In terms of proliferation, when cultured for 0 days, the *γδ*T cells in each group accounted for 3%-5% of the total monocytes, which is consistent with the reported that *γδ*T cells occupied 0.5%-5% of PBMC. After 14 days of culture, the *γδ*T cells in each group accounted for 25%-35% of the total PBMC. Compared with the control group, the expansion multiples of each group were significantly increased. Compared with the control group, the expansion multiples of each group were significantly increased, indicating that Rukang decoction, PHA, and ZOL exert a stimulating effect on the proliferation of *γδ*T cells.

The antitumor mechanism of Chinese medicine has always been an important area of clinical exploration. It is generally believed that Chinese medicine exerts an immunomodulatory effect in the body by regulating T, B lymphocytes, mononuclear macrophages, immune cytokines, dendritic cells, and tumors. Infiltrate lymphocytes and other cellular molecules can exert antitumor immune effects [24]. In particular, the effective ingredients of traditional Chinese medicines are a hot research topic. It has been reported that quercetin can significantly promote the proliferation of *γδ*T cells, the expression of granzyme B, and perforin as well as the ability to kill colon cancer HCT116 cells. The mechanism may be through the signal pathways of p-ERK and p-Akt [25]. Traditional Chinese medicine polysaccharides can produce powerful antitumor immunity by regulating the immune response of *γδ*T cells. For example, astragalus polysaccharide and poria polysaccharide can significantly inhibit tumor growth in tumor-bearing mice and show a dose-dependent characteristic [26]. Mechanism studies found that the ability of *γδ*T cells in the polysaccharide treatment group of traditional Chinese medicine was enhanced. Meanwhile, the secretion of cytokines INF-*γ*, TNF-*α*, and granzyme increased significantly, and the expression of Fas-L on the cell surface was increased.

This experimental study shows that RKY combined with *γδ*T can increase the killing rate of breast cancer MDA-MB-231 cells. Generally, tumor cells are not sensitive to *γδ*T cells alone [27]. Therefore, other drugs are often supplemented to increase the sensitivity of breast cancer cells to *γδ*T cells, which provides an effective way to improve its efficacy. Huang [28] used a naturally occurring polyphenol drug resveratrol combined with *γδ*T cells to act on cancer cells. Studies have proved that resveratrol can downregulate the expression of c-FLIP in breast cancer cells and increase breast cancer cells' response to *γδ*T cells. The sensitivity of *γδ*T cells to MDA-MB-231 breast cancer cells is enhanced. The research of Yuan et al. [29] showed that puerarin can promote the proliferation of human *γδ* T cells and increase the killing activity of *γδ* T cells against liver cancer SMMC-7721 cells. Research conducted by Zheng et al. [25] showed that quercetin can enhance the proliferation of *γδ*T cells and kill the function of colon cancer HCT116 cells in vitro. In addition, the mechanism may be through the p-ERK and p-Akt signaling pathways. Therefore, in the composition of Rukang decoction, it is speculated that quercetin [25], astragalus polysaccharides, tuckahoe polysaccharides [26], and even curcumol [30], coix seed fat [31], and saikosaponin [32] played a coordinated role. Since there are many effective ingredients in compound Chinese medicines with varying contents, the effective working concentrations of these ingredients are different. Moreover, further research on the disassembly of the formula is needed to fully reveal the mechanism of compound Chinese medicine on breast cancer cell proliferation and apoptosis. In short, being supplemented with drugs to enhance the killing effect of *γδ*T cells on tumor cells in adoptive immunotherapy is effective, which provides more efficient strategies and ideas for tumor immunotherapy.

## Figures and Tables

**Figure 1:** Trypan blue staining of each group at day 0 of culture.

**Figure 2:** Trypan blue staining of each group at 14 days of culture.

**Figure 3:** The expansion of *γδ*T cells in each group at day 0 of culture.

**Figure 4:** The expansion of *γδ*T cells in each group at 14 days of culture.

**Figure 5:** The expansion of *γδ*T cells in each group at 0 and 14 days of culture.

**Figure 6:** Flow cytometric detection of *γδ*T cell expansion times in each group.

**Figure 7:** Test results of the *γδ*T cell killing rate in each group.

**Figure 8:** The killing of MDA-MB-231 cells by *γδ*T cells in each group.

**Figure 9:** Test results of the *γδ*T cell killing rate in each group.

**Table 1:** Cell viability of each group detected by trypan blue at day 0 and day 14 in culture (%).

Group	PBMC	RKY	ZOL	PHA	RKY+ZOL	RKY+PHA	ZOL+PHA	RKY+ZOL+PHA
0	100	100	100	100	100	100	100	100
14	100	95	95	90	90	90	95	95

**Table 2:** Expansion results of *γδ*T cells in each group at 0 and 14 days of culture (($\bar{x}\pm s$) %, *n* = 3).

Group	PBMC	RKY	ZOL	PHA	RKY+ZOL	RKY+PHA	ZOL+PHA	RKY+ZOL+PHA
0	3.50 ± 0.72	3.97 ± 0.45	3.99 ± 0.15	4.37 ± 0.24	4.47 ± 0.97	4.59 ± 1.35	3.45 ± 0.40	3.89 ± 0.48
14	4.77 ± 0.78	23.22 ± 2.73	26.4 ± 0.92	28.66 ± 1.43	27.99 ± 1.10	30.21 ± 1.91	32.51 ± 0.74	33.21 ± 0.42
*t*	2.072	12.051	41.641	29.015	27.777	18.972	59.836	79.622
*p*	0.107	<0.001	<0.001	<0.001	<0.001	<0.001	<0.001	<0.001

Note: when cultured for 0 days, the comparison between groups was *F* = 1.093, *p* = 0.412; when cultured for 14 days, the comparison between groups was *F* = 119.917, *p* < 0.001.

**Table 3:** Flow cytometric detection of *γδ*T cell expansion multiples of each group (*n* = 3).

Group	PBMC	RKY	ZOL	PHA	RKY+ZOL	RKY+PHA	ZOL+PHA	RKY+ZOL+PHA
Amplification factor	1.14 ± 0.44	5.25 ± 0.77	5.70 ± 0.89	6.05 ± 1.03	6.21 ± 0.09	6.76 ± 1.46	7.52 ± 1.05	7.97 ± 1.55

Note: comparison between groups *F* = 17.772, *p* < 0.001.

**Table 4:** Flow cytometric detection of *γδ*T cell killing rate in each group (($\bar{x}\pm s$) %, *n* = 3).

Group	PBMC	RKY	ZOL	PHA	RKY+ZOL	RKY+PHA	ZOL+PHA	RKY+ZOL+PHA
Kill rate	1.08 ± 0.03	1.89 ± 0.14	1.22 ± 0.11	1.31 ± 0.09	1.48 ± 0.10	2.02 ± 0.21	2.18 ± 0.27	2.37 ± 0.35

Note: *F* = 20.498, *p* < 0.001.

## Data Availability

The data used to support the findings of this study are available from the corresponding author upon request.
